# Does periodic lung screening of films meets standards?

**DOI:** 10.12669/pjms.326.11267

**Published:** 2016

**Authors:** Songul Binay, Peri Arbak, Alp Alper Safak, Ege Gulec Balbay, Cahit Bilgin, Naciye Karatas

**Affiliations:** 1 Dr. Songul Binay, MD. Department of Chest Diseases, Yildirim Beyazit University, Medical School, Ankara, Turkey; 2 Prof. Dr. Peri Arbak, MD. Department of Chest Diseases, Duzce University, Medical School, Duzce, Turkey; 3 Prof. Dr. Alp Alper Safak, MD. Department of Radiology, Duzce University, Medical School, Duzce, Turkey; 4 Dr. Ege Gulec Balbay, MD. Associate Professor, Department of Chest Diseases, Duzce University, Medical School, Duzce, Turkey; 5 Dr. Cahit Bilgin, MD. Assistant Professor, Department of Chest Diseases, Sakarya University, Medical School, Sakarya, Turkey; 6 Dr. Naciye Karatas, MD. Department of Chest Diseases, Antakya Goverment Hospital, Hatay, Turkey

**Keywords:** Differences among observers, Periodic screening, Occupational health, Pneumoconiosis, Quality of radiography

## Abstract

**Objective:**

To determine whether the workers’ periodic chest x-ray screening techniques in accordance with the quality standards is the responsibility of physicians. Evaluation of differences of interpretations by physicians in different levels of education and the importance of standardization of interpretation.

**Methods:**

Previously taken chest radiographs of 400 workers who are working in a factory producing the glass run channels were evaluated according to technical and quality standards by three observers (pulmonologist, radiologist, pulmonologist assistant). There was a perfect concordance between radiologist and pulmonologist for the underpenetrated films. Whereas there was perfect concordance between pulmonologist and pulmonologist assistant for over penetrated films.

**Results:**

Pulmonologist (52%) has interpreted the dose of the films as regular more than other observers (radiologist; 44.3%, pulmonologist assistant; 30.4%). The frequency of interpretation of the films as taken in inspiratory phase by the pulmonologist (81.7%) was less than other observers (radiologist; 92.1%, pulmonologist assistant; 92.6%). The rate of the pulmonologist (53.5%) was higher than the other observers (radiologist; 44.6%, pulmonologist assistant; 41.8%) for the assessment of the positioning of the patients as symmetrical. Pulmonologist assistant (15.3%) was the one who most commonly reported the parenchymal findings (radiologist; 2.2%, pulmonologist; 12.9%).

**Conclusion:**

It is necessary to reorganize the technical standards and exposure procedures for improving the quality of the chest radiographs. The reappraisal of all interpreters and continuous training of technicians is required.

## INTRODUCTION

Chest X-ray is one of the most commonly used methods in monitoring and evaluating the respiratory health of employees alongside the pulmonary function tests. Technique and quality of chest radiography is of great importance in the diagnosis of occupational lung disease. Hence, according to the guidelines for assessment of pneumoconiosis of the International Labour Office (ILO), chest radiographs are divided into four subgroups based on technical quality from unacceptable to the good.^1^

Especially the poor quality of the radiographs has been shown to increase the inter observer discrepancies in the assessment of pneumoconiosis. It has been observed that the low-dose chest x-ray of the overweight individuals appear to be misinterpreted due to increased thickness of the chest.^2^ It is emphasized that the interpretation of chest radiography with proper techniques is a valuable method in the diagnosis of occupational diseases. Courses for the training of technicians and physicians have been proposed for these purposes.^3^,^4^

In former publications there are contradictory samples about effectiveness of the technical quality of the films on interpretation.^5^-^7^ It is indicated that lack of radiological classification and sample sets are responsible on misinterpretation of Pneumoconiosis rather than the technical quality of the films.

Some of the technical issues concerning the conventional chest radiography are ceased as replaced by digital radiography. Diagnostic accuracy of image can be increased by adjusting the image quality of digital X-ray. The radiation exposure of the patients reduces as well as the overall cost due to lack of X-ray films. Digital images can be archived much more safely. Finally, computer-aided diagnosis can be done by the quantitative analysis of digital radiographic images.^8^ Although, conventional chest radiography is mostly replaced by digital radiography, it is still used for chest screening by some establishments. The ability of evaluating chest radiographs in terms of quality and technical specifications before interpretation is essential for physicians. Physicians should be trained and experienced in this regard. For epidemiological studies (in case of inability of repeating) the technical inadequacies of the films should be recorded in detail.

The aim of our study was to assess the level of compliance of the three readers who are in different disciplines and levels of education (pulmonologist, pulmonologist assistant and radiologist), in the evaluation of chest radiographs taken by mobile X-ray systems in terms of technology and quality.

## METHODS

The study included 404 employees who have periodic chest radiographs in a factory that produces glass run channels in Duzce. They were chosen out of 1600 employees by Simple Random Sampling method. Radiographs were interpreted by faculty members of Department of Radiology (observer 1), and Department of Chest Diseases (observer 2) and also by research fellow of department of Chest Diseases (observer 3). During the interpretation of the chest radiographs; the dose of the films (regular, over or underpenetrated), the adequacy of inspiration, the positioning of patients (symmetrical, right anterior oblique, left anterior oblique), the positioning of scapulae (superimposed to lungs or not) and the apices (visualized in the films or not) mentioned by the observers independently.

Frequency analyses of the data were performed by SPSS 13.0 statistical analysis program. Interobserver discrepancies and (kappa analysis) analysis were performed. Kappa value <0 is accepted as discordant, whereas 0:01 to 0:20 with weak, between 0:21 to 0:40 with a poor, between 0.41-0.60 moderate, 0.61 to 0.80 with good, while those between 0.81-0.99 with perfect concordance.

## RESULTS

The comments of the 3 observers about the films of 404 employees are shown in Fig.1.

**Fig.1:** Comments of the 3 observers about the dose of the films. Difference between radiologist and pulmonologist p = 0.0002, Difference between radiologist and pulmonologist assistant p = 0.0006, Difference between pulmonologist and pulmonologist assistant p = 0.0001,

Pulmonologist (52%) has interpreted the dose of the films as regular more than other observers (radiologist; 44.3%, pulmonologist assistant; 30.4%). The rate of the assessment of the films as over penetrated was higher for the radiologist (45.3%) than others (pulmonologist; 28.5%, pulmonologist assistant; 33.4%). The differences between interpretation of the dose assessments of three observers were statistically significant. The assessment of the films as being inspiratory or expiratory phase by the observers is shown in Table-I.

**Table-I:** Concordance rates of the observers on technique and quality of the films.

		Radiolog –Pulmonolog		Radiolog – Pul. assist		Pulmonolog–Pul. assist	

		Kappa	Agree%	Kappa	Agree%	Kappa	Agree%
Penetration	Normal	0.285	64.1	0.150	59.4	0.332	66.1
	Under	0.474	86.4	0.290	72.2	0.470	77.9
	Over	0.505	76.2	0.581	79.7	0.677	86.1
Taken in inspirium		0.427	86.6	0.406	91.6	0.505	88.6
Position	Symmetric	0.322	65.8	0.471	74.0	0.320	65.6
	Right oblique	0.426	81.4	0.589	85.9	0.492	81.2
	Left oblique	0.507	78.4	0.643	83.6	0.530	80.9
Scapulae excluded		0.851	92.5	0.835	91.8	0.875	93.8
Apices observed		0.545	96.5	0.243	91.3	0.277	92.3
Graph fit into cassette		0.494	80.4	0.510	76.7	0.415	72.0

The frequency of interpretation of the films as taken in inspiratory phase by the pulmonologist (81.7%) was less than other observers (radiologist; 92.1%, pulmonologist assistant; 92.6%). The differences between all three observers, in determining whether the films were taken in inspiratory phase were statistically significant Difference between radiologist and pulmonologist; p = 0.0004, Difference between radiologist and pulmonologist assistant; p = 0.0001, Difference between pulmonologist and pulmonologist assistant; p = 0.0005. The films according to the positioning of the patients are shown in Fig.2.

**Fig.2:** Interpretation According to the positioning. Difference between radiologist and pulmonologist; p = 0.0003, Difference between radiologist and pulmonologist assistant; p = 0.0002, Difference between pulmonologist and pulmonologist assistant; p = 0.0002,

The rate of the pulmonologist (53.5%) was higher than the other observers (radiologist; 44.6%, pulmonologist assistant; 41.8%) for the assessment of the positioning of the patients as symmetrical. The films were interpreted as left anterior oblique more frequently by the radiologist (38.1%), than other observers (pulmonologist; 23.5% pulmonologist assistant; (32.2%). In terms of the positioning of the films, differences between three observers were statistically significant.

The evaluations of the observers according to the positioning of the scapulae are shown in Table-I. The exclusion of the scapulae is mentioned most frequently by pulmonologist assistant (pulmonologist assistant; 55.9%, radiologist; 53.7%, pulmonologist; 52.7%). The differences for specifying the exclusion of the scapulae between three observers were statistically significant. Difference between radiologist and pulmonologist; p = 0.0003, difference between radiologist and pulmonologist assistant; p = 0.0005, difference between pulmonologist and pulmonologist assistant; p = 0.0009,

The interpretations of the observers for the visualization of apices of the lungs can be seen in Table-I. The frequency of indicating the visualization of the apices was the least for pulmonologist assistant (pulmonologist assistant; 92.3%, radiologist; 95.5%, pulmonologist; 96.5%). There were statistically significant differences in concerning the visualization of the apices between three observers. Difference between radiologist and pulmonologist; p = 0.0001, difference between radiologist and pulmonologist assistant; p <0.0001, difference between pulmonologist and pulmonologist assistant; p = 0.0002,

The interpretations of the observers whether the lungs were included on films are also shown in Table-I. The fitting of the lungs on films was least mentioned by pulmonologist assistant (pulmonologist assistant; 55%, radiologist; 75.7%, pulmonologist; 72%). There were statistically significant differences in the detection of lungs fitting on the films between the three observers. Difference between radiologist and pulmonologist; p = 0.0001, difference between radiologist and pulmonologist assistant; p = 0.0002, difference between pulmonologist and pulmonologist assistant; p = 0.0001,

Interobserver concordance rates for the technique and quality of the films are shown in Table-I. There was perfect concordance between observers one and two on underpenetrated films whereas there was perfect concordance between observers two and three on overpenetrated films. Observer 1 and 3 were moderately concordant about the films that the dose determined to be regular. All the other interpretations were in good concordance for the dose levels of the films. The interpretations on level of inspiration, exclusion of the scapulae and visualization of the apices were in perfect concordance.

Concordance among all observers on films with the right anterior oblique position was perfect. Concordance for left anterior oblique projections was perfect between observers one and three and between observers two and three had perfect. All the other interpretations on positioning were with good concordance.

The interpretations on fitting of the whole lungs to films were in perfect concordance for observer one and two. All the other interpretations about the fitting of the lungs to films were with good concordance. The interpretations of observers for presence of parenchymal findings are shown in Fig.3.

**Fig.3:** Interpretations on the presence of parenchymal findings. Difference between pulmonologist and radiologist; p = 0.002, Differences between pulmonologist and radiologist; p = 0.002, Differences between pulmonologist assistant and radiologist; p = 0.006

Parenchymal findings were mostly mentioned by pulmonologist assistant (15.3%) with respect to others (radiologist, 2.2%, pulmonologist; 12.9%). The differences between pulmonologist and radiologist (p = 0.002) as well as pulmonologist assistant and radiologist (p = 0.006) were statistically significant for reporting parenchymal findings.

Interobserver concordance rates of the radiological findings were perfect between radiologist and pulmonologist (kappa: 0.131, agreement rate: 87.4%), pulmonologist assistant and radiologist (kappa: 0.106, agreement rate: 84.9) whereas, good between pulmonologist assistant and pulmonologist (kappa: 0.021, agreement rate: 76.2 %).

## DISCUSSION

The effectiveness of early diagnosis of chest radiography in the detection of occupational lung diseases is decreasing due to the technical quality insufficiencies. Therefore, the increase in the quality of the radiographs requires the improvement of the radiographers’ performance and technical infrastructure. Staff qualifications and responsibilities are clearly defined by the NIOSH Guide. Medical physicists might be employed for imaging facilities to ensure the reliability of the adequacy of pneumoconiosis classification. The medical physicist should be qualified or familiar with the quality assurance programs of the facilities and in assessing the performance of radiological equipment. He/she must be licensed, approved or certificated by the authorized boards and must have the master degree on related fields with continuing education and experience. Radiographers should be trained on the software and equipment used in the radiology department or should be certified or experienced to implement the general radiographic procedures established by the authorized board. The physicians who are using ILO classification should have appropriate education and experience including regular digital chest X-ray and certificated by the boards of pulmonary, occupational medicine or radiology and / or should be competent in the assessment of pneumoconiosis radiographs as reader B by NIOSH.^9^

In addition, features of the interpreters are stated clearly by the NIOSH guide. According to this; medical diagnosis, medical imaging, chest radiography classification for screening, government programs and disapproval procedures must be performed by a physician who is experienced and has the privilege of using the ILO International Radiography Classification with the allegiance of serving to patient, worker and community welfare. Interpreters should be aware of four components necessary for correct classification of pneumoconiosis. These components are; 1) appropriate methods for image acquisition and display, 2) interpreters’ competence, 3) ethical allegiance to classification, 4) using suitable radiological methods. Interpreters must have the ability of continuous experience, education, and compatibility with the participation of NIOSH-B reader approval program.^9^

In this study, dose assessment rates of the films were found to be regular between 30.4-52% by the observers. In this case, the speed of being in regular dose of the films in periodic screening remained at 50%. These data suggested that the film quality should be improved in periodic screenings. Rega and Morgan have mentioned in their study about the film quality that the determination rates for suitable films were between 79.8- 98.2% among three radiologist and one epidemiologist.^7^ In both studies common point was the inconsistencies between interpreters. One study revealed that the radiologists during the evaluation of pediatric chest X-ray; due to insufficient clinical data of their patients, they showed a tendency to report more abnormal findings in order to avoid misdiagnosis and malpractice charges.^10^ In our study, pulmonologist (52%) have mentioned the films as regular more often than radiologist. Also assessment rate of films as overpenetrated by the radiologist (45.3%) was higher than the pulmonologist.

Regina and colleagues have observed a significant effect of the film quality on radiographic categorization of coal workers pneumoconiosis.^11^ There was a marked tendency for further evaluation for underpenetrated films whereas the opposite was also valid for overpenetrated films. Although it may seem like there’s tendency for all interpreters, some were more impressed than others. This was valid for both under and over penetrated films and experienced interpreters are less affected. Cimrin and his colleagues have mentioned that 50% of the films of the workers in a lignite plant were observed to be poor and 9% was very poor in terms of technical quality.^12^ In our study the rates of interpreting the exclusion of the scapulae by all observers were 52.7 to 55.9%. The detection rates of indicating the films as symmetric were 41.8 to 53.5 whereas for inclusion of all lungs were 55 to 75.7%.

According to our results, almost 50% of the films were over or underpenetrated, the exclusion of the scapula was acceptable for 45% of the films, symmetry could not be achieved in almost 45% of the films and the average of the film rates including the whole lungs remained at 70%.

Technical quality has very important influences especially on the pneumoconiosis classification. Usually underexposure leads for a higher; overexposure leads for a lower category in ILO classification. The factors for the differences in the interpretation of films between the observers depends on different levels of medical education, difficulty in getting previous radiographs and clinical data and even the conditions of reading rooms. Training in film reading and improvement of experience reduce the differences between readers.^13^

There are publications on failures of interpretation of chest radiographs by emergency physicians, general practitioners and anesthesiologists. The conditions for becoming a successful reader for chest radiography are listed as level of education, field of education, willing to do pulmonology training.^14^ It is also important not to interpret a normal chest x-ray as abnormal. Misdiagnosis may lead to erroneous medical decisions.^15^,^16^

## CONCLUSION

Our study consisted of a group with unexpected pneumoconiosis. The perfect concordances among observers determined on technical quality of the films were on respiratory phases, the exclusion of the scapulae and visualization of apices, respectively. It is considered that to achieve better concordance on exposure doses, symmetry of the chest and inclusion of the whole lungs, the observers should be informed for standardization. As a result; the interpretation of the radiographs by three different observers, taken for periodic screening of a group of workers with unexpected pneumoconiosis; in almost 50% of the films, technical quality of the films and the exposure doses were observed to be insufficient. Readers are determined to show significant differences in interpreting the technical and quality characteristics of the films. A national program is needed to be developed for the elimination of the discrepancies between exposure, positioning techniques and interpretation of radiographs especially in periodic screening.
